The article "Pharmacological Effect of Panax notoginseng Saponins on Cerebral Ischemia in Animal Models" was published in 2022. Journal: Biomed Res Int.

# Pharmacological Effect of *Panax notoginseng* Saponins on Cerebral Ischemia in Animal Models

**DOI:** 10.1155/2022/4281483

**Published:** 2022-08-04

**Authors:** Chao Dong, Jiawei Li, Ming Zhao, Lin Chen, Xiaochen Zhai, Lingling Song, Jin Zhao, Qiang Sun, Jie Wu, Xiaolu Xie

**Affiliations:** ^1^Department of Pharmacology, School of Basic Medical Science, Xi'an Jiaotong University Health Science Center, Xi'an, Shaanxi 710061, China; ^2^Key Laboratory of Environment and Genes Related to Disease, Ministry of Education of the People's Republic of China, China; ^3^Department of Pharmacy, The First Affiliated Hospital of Xi'an Medical University, Xi'an 710077, China; ^4^Department of Cardiology, The First Affiliated Hospital of Medical College, Xi'an Jiaotong University, Xi'an, Shaanxi 710061, China

## Abstract

*Panax notoginseng* saponins (PNS), bioactive compounds, are commonly used to treat ischemic heart and cerebral diseases in China and other Asian countries. Most previous studies of PNS have focused on the mechanisms underlying their treatment of ischemic cardiovascular diseases but not cerebral ischemic diseases. This study sought to explore the pharmacological mechanisms underlying the effectiveness of PNS in treating cerebral ischemic diseases. Different experimental cerebral ischemia models (including middle cerebral artery occlusion (MCAO) and the blockade of four arteries in rats, collagen-adrenaline-induced systemic intravascular thrombosis in mice, thrombosis of carotid artery-jugular vein blood flow in the bypass of rats, and hypoxia tolerance in mice) were used to investigate the mechanisms underlying the actions of PNS on cerebral ischemia. The results indicated that (1) PNS improved neurological function and reduced the cerebral ischemia infraction area in MCAO rats; (2) PNS improved motor coordination function in rats with complete cerebral ischemia (blockade of four arteries), decreased Ca^2+^ levels, and ameliorated energy metabolism in the brains of ischemia rats; (3) PNS reduced thrombosis in common carotid artery-jugular vein blood flow in the bypass of rats; (4) PNS provided significant promise in antistroke hemiplegia and hypoxia tolerance in mice. In conclusion, PNS showed antagonistic effects on ischemic stroke, and pharmacological mechanisms are likely to be associated with the reduction of cerebral pathological damage, thrombolysis, antihypoxia, and improvement in the intracellular Ca^2+^ overload and cerebral energy metabolism.

## 1. Introduction

Cerebral ischemic stroke is a major global health problem and a leading cause of death and long-term adult disability [1, 2]. This disease continues to be a devastating disorder, and cerebral ischemia/reperfusion-elicited tissue injury contributes to morbidity rates of 30% and 50% in one month and one year, respectively [1, 3]. Cerebral ischemic stroke manifests from the disruption of cerebral blood supply because of a blockade in a specific brain areas by artery stenosis or thrombosis, leading to the disorder of energy supply and brain tissue hypoxic-ischemic death, a chief cause of disability and third leading cause of death worldwide following cardiovascular diseases and cancer [4]. Currently, the drug used for cerebral ischemic stroke is mainly dedicated to therapies such as thrombolysis, improvement in microcirculation, restoration of the blood supply to the ischemic area, anticoagulation, reduction of blood viscosity, neuroprotection, reduction of ischemic cerebral edema, and the prevention and treatment of complications [5, 6]. In addition to synthetic chemicals, many natural products and herbal extracts, such as oleuropein, pomegranate extract, and shikonin [6–8], have demonstrated activity in treating cerebral ischemia.

*Panax notoginseng* saponins (PNS), bioactive compounds with a range of medical applications, are extracted from the roots and rhizomes of *Panax notoginseng* (Burk.) F.H. Chen [9]. Lines of evidence have demonstrated that PNS has extensive beneficial effects on cardiovascular system diseases [10–14]. Recently, a few reports have shown that PNS could also effectively treat cerebral ischemic diseases [15–17]. However, its action mechanisms on cerebral ischemic diseases are primarily based on knowledge derived from studies of PNS used to treat cardiovascular ischemic diseases. The discrepancy in physiological conditions between cardiac tissue and cerebral tissue, particularly due to the blocking action of the blood–brain barrier (BBB), makes the two tissue types react differently to many medications so that the therapeutic efficacy is not the same. Zhang et al. reported that PNS demonstrated the clearly neuroprotective effect against ischemia/reperfusion injury (IRI). They identified 9 transcription factors that were the key targets in the protection of PNS against cerebral IRI [16]. Using an animal cerebral ischemic model, Hu et al. found that PNS improves the protective effect for the cerebral injury caused by ischemia/reperfusion (IR) [17]. Although these studies have made an exploratory attempt to explain the action of PNS on cerebral ischemic stroke, the underlying mechanisms by which PNS are effective in treating cerebral ischemic diseases remain unclear. The present study sought to explore the mechanisms by which PNS effectively treat cerebral ischemic diseases using cerebral infarction and hypoxia animal models. The pharmacological effects revealed herein will improve understanding of the mechanisms of PNS in the clinical treatment of cerebral ischemic disease.

## 2. Materials and Methods

### 2.1. Animals

Male Sprague–Dawley rats (180-220 g) and male Institute of Cancer Research (ICR) mice (19-32 g) were provided by the Experimental Animal Center of Xi'an Jiaotong University (Xi'an, Shaanxi, China). Experimental animals were maintained at 22°C and 55% humidity with a 12-h light/12-h dark cycle and were allowed access to food and water *ad libitum*. All the procedures were performed in accordance with standard guidelines as described in the Guide for the Care and Use of Laboratory Animals (US National Institutes of Health 85-23, revised 1996). All the animal experimental protocols were approved by the Experimental Animal Committee of Xi'an Jiaotong University.

### 2.2. Reagents

Triphenyl tetrazolium chloride was purchased from China Pharmaceutical-Shanghai Chemical Reagent Co., Ltd. Collagen was purchased from Sigma (St. Louis, MO, USA). Adrenaline HCl injection was purchased from Wuhan Pharmaceutical Group Co., Ltd. (Wuhan, Hubei, China). PNS (dissolved in 5% glucose solution to yield the desired concentrations) were kindly provided by Xi'an Wanlong Pharmaceutical Co., Ltd. (Xi'an, Shaanxi, China).

### 2.3. Experimental Design

#### 2.3.1. Cerebral Ischemia in Rats Subjected to Middle Cerebral Artery Occlusion (MCAO) [18]

Male rats were anesthetized by intraperitoneal injection of 40 mg/kg of 4% sodium pentobarbital. Subsequently, the right common, internal, and external carotid arteries of rats were exposed. Except for the sham-operated (SO) group, the internal and external carotid arteries of the remaining rats were ligated. A small incision was made in the internal and external carotid bifurcation of the right common carotid artery, and a round-headed 0.26-mm nylon thread was inserted into the right common carotid artery and slowly moved to the distal end approximately 18.5 ± 0.5 mm from the bifurcation until slight resistance was felt. Next, the internal carotid artery was ligated, and the skin was sutured with nylon thread. Subsequently, fifty rats were randomized into five experimental groups (*n* = 10 rats/group). Rats in each group were intravenously injected with the corresponding drugs at 9.13 ml/kg as follows: (1) SO group, in which surgical preparation was conducted without internal carotid artery ligation and rats were treated with 5% glucose solution (9.13 ml/kg body weight); (2) MCAO group, MCAO rats were treated with 5% glucose solution (9.13 ml/kg body weight); (3) low-dose PNS-treated group, MCAO rats were treated with PNS (18.3 mg/kg body weight); (4) middle-dose PNS-treated group, MCAO rats were treated with PNS (36.5 mg/kg body weight); (5) high-dose PNS-treated group, MCAO rats were treated with PNS (73 mg/kg body weight). During surgery, room temperature was maintained at 24 ± 0.5°C, and the animals were incubated to maintain a rectal temperature of 37.0 ± 0.5°C both intraoperatively and postoperatively. Twelve hours after surgery, the corresponding drugs were intravenously given to each group of rats again at the same dosage.

Twenty-four hours after surgery, the single-blind method was used to conduct a neurological assessment according to the Bederson score standard [19], where the higher the score was, the more serious the behavioral disorder was. Following neurological assessment, the rat brains were removed without the olfactory bulb, cerebellum, and lower brainstem to assess the cerebral infarction area. The brains were placed in ice brine for 10 min and then cut into five 2-mm-thick slices. Every slice was rapidly placed into 2% triphenyl tetrazolium chloride (TTC) phosphate buffer solution and incubated for 30 min at 37°C in the dark; the slices were turned once every 7-8 min during this period. Normal brain tissue was stained deep red, leaving the infarct tissues unstained. A digital camera was used to image bilateral brain slices, and images were analyzed using the Scion Image Beta 4.0.2 software to calculate the infarction area and brain area. The ratio of the total infarct area and brain area for the 5 brain slices of each rat was adopted as the cerebral ischemic infraction area ratio (%).

#### 2.3.2. Cerebral Ischemia in Rats Subjected to Four-Vessel Occlusion [20]

Fifty male rats were randomized into five experimental groups (*n* = 10 rats/group) as follows: (1) SO group, in which surgical preparation was conducted without four artery ligation and the rats were treated with 5% glucose solution (9.13 ml/kg body weight); (2) ischemia model group, in which the rats were treated with 5% glucose solution (9.13 ml/kg body weight); (3) low-dose PNS-treated group, in which ischemia model rats were treated with PNS (18.3 mg/kg body weight); (4) middle-dose PNS-treated group, in which ischemia model rats were treated with PNS (36.5 mg/kg body weight); (5) high-dose PNS-treated group, in which ischemia model rats were treated with PNS (73 mg/kg body weight). The rats were anesthetized by inhalation of ether, fixed in the supine position. An incision was made in the dorsal midline occipital between the first and second cervical vertebrae, and the transverse process of the first cervical vertebra was exposed under a microscope. Immediately thereafter, the left and right transverse holes were found, and then a 0.5-mm-diameter electric coagulation device was inserted into the two holes to burn the bilateral vertebral artery in all the rats except in the SO group, causing permanent occlusion. Immediately, an incision was made in the middle of the neck, bilateral common carotid arteries were exposed, and reserve lines were set under each side of the bilateral common carotid arteries under sterile conditions. Next, the wound was sutured. During surgery, room temperature was maintained at 24 ± 0.5°C, and the animals were incubated to maintain a rectal temperature of 37.0 ± 0.5°C both intraoperatively and postoperatively.

Immediately and 24 h after surgery, rats in all groups were intravenously injected with the corresponding drugs. Thirty minutes after the second injection, the inclined plane method was used to test the motor coordination function of animals as described previously [21]. Each rat was placed on a 0°-angled 40 × 30 cm^2^ inclined smooth plane in the upheaded position (head-up orientation), and the angle of the inclined plane was increased at a rate of 2°/sec from 0° to 90°. The maximum angle was then recorded at the moment when a limb of the rat slipped to maintain body position. The test was performed three times and averaged. Each trial was performed after a 1-minute interval. Subsequently, the neck suture was removed from all the rats except those in the SO group, and the bilateral common carotid arteries were clamped with small clips (four vessel occlusions) for 30 min. Next, the clips were released to allow reperfusion of the cerebral ischemia area via common carotid arteries. Three hours later, rats in all groups were decapitated, and the heads were rapidly placed in liquid nitrogen for 15 min. The whole brain of each rat was then removed and weighed to calculate the brain index (g/(100 g weight)) to examine cerebral edema. The whole brain was placed in 2 ml of Tris-HCl buffer solution (0°C, pH 7.4) and homogenized for 30 s at 700 rpm before adding another 6 mL of Tris-HCl buffer. To analyze energy metabolism, the samples were then centrifuged for 30 min at 3000 rpm at 4°C, and the supernatants were collected to determine the concentrations of lactic acid (LA), adenosine triphosphate (ATP), phosphocreatine (PCr), free fatty acids (FFAs), and Ca^2+^.

#### 2.3.3. Collagen-Adrenaline-Induced Thrombosis in Mice

Forty-eight male mice were randomized into the following four groups (*n* = 12 mice/group) and intravenously injected with the corresponding drugs: (1) thrombosis model group, in which the mice were injected with 5% glucose solution (13.1 ml/kg body weight); (2) low-dose PNS-treated group, in which the mice were treated with PNS (26.2 mg/kg body weight); (3) middle-dose PNS-treated group, in which the mice were treated with PNS (52.4 mg/kg body weight); (4) high-dose PNS-treated group, in which the mice were treated with PNS (104.8 mg/kg body weight). The mice in each group were intravenously injected with 13.1 ml/kg of the corresponding drugs. Fifteen minutes later, a mixture of collagen (7.5 mg/kg) and adrenaline (300 *μ*g/kg) was injected into the tail vein of mice in each group to induce systemic thromboembolism as described previously [22]. The number of dead mice within 5 min and the number of hemiplegic (paralyzed) mice within 15 min in each group were recorded.

#### 2.3.4. Carotid Artery-Jugular Vein Thrombosis in Rats [23]

Forty male rats were randomized into the following groups (*n* = 10 rats/group) and intravenously injected with the corresponding drug: (1) thrombosis model group, in which the rats were treated with 5% glucose solution (9.13 ml/kg body weight); (2) low-dose PNS-treated group, in which the thrombosis model rats were treated with PNS (18.3 mg/kg body weight); (3) middle-dose PNS-treated group, in which the thrombosis model rats were treated with PNS (36.5 mg/kg body weight); (4) high-dose PNS-treated group, in which the thrombosis model rats were treated with PNS (73.0 mg/kg body weight). After anesthetization by intraperitoneal injection of 4% sodium pentobarbital (40 mg/kg body weight), the rats were fixed in the dorsal position, and the trachea was intubated. The common carotid artery and left external jugular vein were simultaneously separated. Next, a 7-cm-long shunt comprising three sections of polyethylene plastic pipe and including a built-in, preweighed 5-cm length of No. 4 surgical thread was filled with heparin saline (50 U/ml), and one end was inserted into the left external jugular vein before ligating the vein. Heparin saline (50 U/ml) was also injected into the other end of the casing at a dosage of 50 U/kg body weight before insertion into the right common carotid artery and ligation. Immediately after the operation, the rats in all the groups were intravenously injected with the corresponding drugs in each group one time. Five minutes after injection, the right common carotid artery was released so that blood could flow through the polyethylene pipe into the left external jugular vein. Fifteen minutes later, blood flow was again interrupted, and the surgical thread was quickly removed and weighed. The thrombus weight is equal to the wet weight of the surgical thread subtracted by its dry weight, and the formula for the rate of thrombosis inhibition is as follows:

(1) $$\begin{array}{c} \text{Thrombus inhibition }\left(\%\right)=\frac{\text{Control group thrombus weight}-\text{Experimental group thrombus weight}}{\text{Control group thrombus weight}} \end{array}$$

#### 2.3.5. Hypoxia Tolerance Ability in Mice

Forty male mice were randomized into four groups (*n* = 10 mice/group): (1) hypoxia group, in which the mice were treated with 5% glucose solution (13.1 ml/kg body weight); (2) low-dose PNS-treated group, in which the mice were treated with PNS (26.2 mg/kg body weight); (3) middle-dose PNS-treated group, in which the mice were treated with PNS (52.4 mg/kg body weight); (4) high-dose PNS-treated group, in which the mice were treated with PNS (104.8 mg/kg body weight). The mice in all the groups were intravenously injected once with 13.1 ml/kg of the corresponding drugs. Fifteen minutes after administration, each mouse was placed in a 250-ml jar sealed airtight with a lid and petrolatum as described previously [24]. The time from when the mouse was sealed in the jar to its death was recorded and adopted as the hypoxia tolerance time of mice resistant to hypoxia.

### 2.4. Statistical Analysis

All continuous variables were presented as means ± standard deviation (SD), with the number of experiments shown in parentheses. Statistical comparisons were evaluated using one-way analysis of variance (ANOVA) with the Newman–Keuls *post hoc* test, as appropriate. Categorical variables were evaluated by *χ*^2^ test. A *P* < 0.05 was considered statistically significant.

## 3. Results

### 3.1. PNS Reduce the Cerebral Ischemic Infarction Area and Ameliorate Neurocoordination in MCAO Rats

Representative TTC staining images of coronal sections of rat brain in each group after MCAO are shown in Figure 1(a). Similar to a previous study [18], the ischemic infarction area (in white) was mainly localized to cortical regions. The ratios of the ischemic infarction area in the middle- and high-dose PNS-treated groups were 19.93 ± 3.86% (*n* = 10) and 25.80 ± 5.34% (*n* = 10), respectively, which were significantly (*P* < 0.01) lower than those in the MCAO model group (35.80 ± 6.17, *n* = 10) (Figure 1(b)). These results suggest that PNS reduce cerebral infarction induced by MCAO in a dose-dependent manner.

Neurological deficit scoring is an important index of evaluation to diagnose and heal cerebral ischemia [19]. The bar graphs in Figure 1(c) show that the neurobehavioral scores of rats were 9.5 ± 0.7 (*n* = 10), 8.90 ± 0.99 (*n* = 10), 8.50 ± 1.18 (*n* = 10), and 7.9 ± 0.88 (*n* = 10) in the MCAO model group, low-dose, middle-dose, and high-dose PNS-treated groups after 24 h of cerebral ischemia, respectively. Compared with the score in the MCAO model group, those in the middle- and high-dose PNS-treated groups were significantly (*P* < 0.05 or *P* < 0.01) lower, indicating that PNS ameliorate the neurocoordination function of MCAO rats.

### 3.2. PNS Improve Motor Coordination Function in Focal Cerebral Ischemia Rats and Energy Metabolism in Rats Subjected to Cerebral Ischemia/Reperfusion Injury

The average maximum angle, at which rats slipped down from the inclined smooth plane, reflects the damage to muscle strength and brain nerve function after bilateral vertebral arteries were occluded (Figure 2(a)). The average maximum angles of the SO group, ischemia model group, and three PNS-treated groups (including low-dose, middle-dose, and high-dose) were 65.67 ± 7.37, 31.84 ± 1.65, 32.43 ± 2.69, 34.01 ± 3.26, and 40.99 ± 3.34 (*n* = 10 rats/group), respectively. The rats in the three PNS-treated groups achieved larger average maximum angles than those in the ischemia model group, with a very significant (*P* < 0.01) difference between the high-dose PNS-treated group and ischemia model group. These results suggest that abnormal motor function caused by neurologic deficits in ischemic rats is improved by PNS.

After the bilateral common carotid arteries were also occluded (four vessel occlusion) for 30 min, the ischemic cerebral tissues of rats were reperfused for 3 hours. Next, the whole brain of each rat was removed to check tissue metabolites. The levels of LA, FFA, and Ca^2+^ in cerebral tissues of the PNS-treated group rats were lower than those in the ischemia model group rats, while the ATP and PCr levels were higher (Table 1). Among these bioactive substances in the rat brain, the LA, FFA, ATP, PCr, and Ca^2+^ levels in the brains of high-dose PNS-treated group rats, as well as the FFA, ATP, PCr, and Ca^2+^ levels in the brains of middle-dose PNS-treated rats, were significantly (*P* < 0.05 or *P* < 0.01) different from those in the brains of ischemia model group rats. Thus, PNS could antagonize the impairment of both brain nervous tissues and cerebral energy metabolism caused by cerebral ischemia. Regarding the cerebral index, although a decrease was found in each PNS-treated group, no significant difference was observed to be related to the cerebral index compared with that in the ischemia model group (Figure 2(b)).

### 3.3. PNS Decrease Systemic Thromboembolism Induced by Collagen-Adrenaline in Mice

Thromboembolism is the most common cause of ischemic stroke. We assessed the effect of PNS on systemic thromboembolism in mice. After the mice were intravenously injected with a mixture of collagen (7.5 mg/kg) and adrenaline (300 *μ*g/kg) to form systemic intravascular thrombosis, both the number of hemiplegic (paralyzed) mice within 15 min (Figures 3(a) and 3(b)) and the number of dead mice within 5 min (Figures 3(c) and 3(d)) in each PNS-treated group were fewer than those in the thrombosis mode. The number of hemiplegic mice in the middle-dose PNS-treated group as well as the number of dead and hemiplegic mice in the high-dose PNS group exhibited significant differences (*P* < 0.05 or *P* < 0.01) relative to those in the thrombosis model group, suggesting the inhibition of systemic intravascular thrombosis by PNS.

### 3.4. PNS Decrease Thrombosis in Common Carotid Artery-Jugular Vein Blood Flow Bypass in Rats

To further observe the inhibitory effect of PNS on thrombus formation, the arteriovenous (AV) shunt thrombosis rat model was employed as previously described [23]. The thrombus weight formed in the common carotid artery-external jugular vein blood flow bypass in the three PNS-treated (low-dose, middle-lose, and high-dose) groups were 14.56 ± 2.81 mg (*n* = 10), 11.41 ± 1.94 mg (*n* = 8), and 10.64 ± 2.15 mg (*n* =10), respectively, all of which were significantly (*P* < 0.01) lighter than that (22.93 ± 3.74 mg; *n* = 10) in the thrombosis model group (Figure 4). The thrombosis inhibition rates in all the PNS-treated (low-dose, middle-dose, and high-dose) groups were 36.5%, 47.9%, and 53.6% (Figure 4 inset), respectively. The inhibitory action of PNS on thrombus formation shows a typical dose-dependent response.

### 3.5. PNS Increase Hypoxia Resistance Ability in Mice

Cerebral ischemia inevitably leads to hypoxia in the brain that is highly sensitive to changes in oxygen concentration because of a high intrinsic oxygen consumption rate. In the present study, mice were placed in a sealed jar to examine the effect of PNS on hypoxia resistance. The hypoxia tolerance time of mice in the PNS-treated groups (the time values of low-dose, middle-dose, and high-dose groups were 25.72 ± 4.33, 28.13 ± 4.73, and 28.50 ± 5.43 seconds, respectively; *n* = 10 mice/group) was longer than that (23.41 ± 3.67 seconds, *n* = 10) of mice in the hypoxia model group, with middle-dose and high-dose PNS-treated groups showing a significant (*P* < 0.05) difference over the hypoxia model group (Figure 5).

## 4. Discussion

In the present study, experimental ischemia animal models were used to explore the mechanisms underlying the protective effect of PNS on cerebral ischemia. PNS reduced the cerebral infarction scope, decreased the intracellular Ca^2+^ levels, and improved neurocoordination function and cerebral energy metabolism in cerebral ischemia rats. Additionally, PNS attenuated thrombosis and increased hypoxia resistance in animals. These findings strongly suggest that the protective effects of PNS on cerebral ischemic diseases involve various pharmacological actions, including reduced cerebral pathological damage, thrombolysis, and antihypoxia and improved intracellular Ca^2+^ overload and cerebral energy metabolism.

A common cause of ischemic stroke is occlusion of the middle cerebral artery, which supplies oxygen and nutrients to sensory and motor areas. Occlusion of this artery is commonly associated with motor and sensory dysfunction [1]. In the present study, PNS significantly improved the neurological function of MCAO rats (Figure 1(c)) and increased the average maximum angle at which cerebral ischemia rats (subjected to occlusion of the bilateral vertebral artery) slipped down from the inclined smooth plane (Figure 2(a)). The neurological abnormalities in posture, hemiparesis, muscle weakness, and total score of neurologic examination were all reduced in PNS-treated rats, suggesting that PNS have the function of improving neurological deficit and coordination ability in local cerebral ischemia. Previously, Ning et al. showed that PNS have neuroprotective effects in a rat model of acute spinal cord IRI [25], a finding that is consistent with our study and provides strong support for our experimental results because neurons in the spinal cord are also responsible for motor coordination. Sensorimotor dysfunction is a well-known sequela of lesions of the frontal cortex and striatum in cerebral ischemia rats, and the severity of neurological deficits has been confirmed to be correlated with the size of the infarction area in the cortex. Compounds such as MK-801 and N-methyl-D-aspartic acid receptor (NMDA) receptor antagonists have demonstrated neuroprotective effects by decreasing the infarction size in parallel with the improvement in behavioral deficits [26, 27]. Similar to these previous findings, TTC staining images of coronal sections of MCAO rat brains (Figure 1(a)) showed that PNS substantially reduced the cerebral infarction area in a dose-dependent manner, indicating that the changes in neurological function caused by PNS in local cerebral ischemia rats were supported by the histologic amelioration of the cortex and basal ganglia. However, we failed to observe significant changes in the cerebral index between PNS-treated rats and ischemia model rats. This finding might indicate that PNS, within the dose range we used, did not remarkably affect ischemic cerebral edema. The BBB, serving as a protective semipermeable membrane for the central nervous system, not only prevents harmful substances from entering the brain but also keeps many medications out of the central nervous system. PNS improved neurological deficits and reduced the cerebral infarction area of local cerebral ischemia rats, implying that PNS crossed the BBB and reached the brain with efficacy.

Most ischemic strokes are thromboembolic in origin, with common sources of embolism in the cerebral vasculature [1, 2]. For acute thromboembolic stroke, early thrombolysis and blood reperfusion are standard therapies for all eligible patients, which can salvage hibernating ischemic penumbra and reduce the risks of additional damage, such as hemorrhagic transformation, oxidative stress, and neuronal functional disorders. In the present study, PNS not only reduced the mortality and hemiplegic rates of systemic thromboembolism mice caused by intravenous injection of a mixture of collagen and adrenaline but also inhibited thrombus formation in common carotid artery-external jugular vein blood flow bypass in rats. These results suggest that PNS have antithrombotic effects that are extremely beneficial to ameliorate blood circulation and the oxygen supply in infarction areas, representing one of the most important pharmacological mechanisms for the efficacy of PNS against cerebral ischemia. Abnormal platelet aggregation and thrombosis are critical factors that cause cerebral ischemia and cerebral infarction. Intravenous injection of a mixture of collagen-adrenaline causes platelet aggregation, leading to systemic thromboembolism and even death by extensive obstruction of microcirculation in vital organs [28]. It should be noted that the collagen-adrenaline-induced thromboembolism is extensive in the mice. Therefore, we cannot exclude the possibility that the paralysis of mice caused by the collagen-adrenaline was not restricted to the transient ischemic attack, but may also be due to the lack of blood perfusion in muscle or alterations not pertaining to the damage of central nervous system. Shen et al. reported that PNS inhibited platelet aggregation induced by thrombin, increased the expression of peroxisome proliferator-activated receptor *γ* protein, and upregulated the phosphatidylinositol 3 kinase/protein kinase B/endothelial nitric oxide synthase pathway in rat [29]. Their finding supports our data that PNS have antithrombotic effects and provides a reasonable mechanistic explanation for our experimental results.

Continuous availability of ATP is essential to maintain normal neuronal functions [2]. When this supply is interrupted, neurons can no longer maintain their transmembrane electrochemical gradient, resulting in the impairment of neuronal functions and catastrophic energy failure in the brain. Numerous clinical observations and animal experimental studies have demonstrated that cerebral hypoxia/ischemia results in substantial declines in ATP and its energy-reserve PCr in all affected areas, usually coinciding with histopathological abnormalities of widespread ischemic cells [30, 31]. Changes in these energy-related metabolites reflect cerebral energy deficiency, which is a crucial contributor to the ultimate brain damage and neurologic compromise. PNS increased the ATP and PCr levels in brain tissue, concomitantly improved neurological deficits, and reduced the cerebral infarction scope in ischemic rats. These data suggest that the improved action of PNS on energy metabolism is involved in its neuroprotective mechanisms against cerebral ischemic damage.

When hypoxia/ischemia occurs, the availability for aerobic energy production through oxidative phosphorylation is diminished, but anaerobic metabolism in fermentation becomes the primary route by which energy is supplied to the tissues, along with a large quantity of the byproducts lactic acid and FFA [31–33]. At this point, lactic acidosis occurs because of the excess lactic acid accumulated under hypoxic conditions, causing cellular injury through multiple pathways, including enhancement of intracellular calcium influx and the secondary release of large amounts of calcium from intracellular stores. Consequently, intracellular calcium overload activates several calcium-dependent processes, such as the activation of neuronal nitric oxide synthase with consequent free radical production and decreased ATP production and the initiation of cell death processes, including apoptosis, necrosis, and autophagy [2]. Additionally, FFAs, produced by calcium-mediated increases in phospholipase activity and consequent degradation of membrane phospholipids, cause further neuronal injury and aggravate regional blood circulation, platelet function, and free radical damage [32, 33]. In the present study, PNS attenuated cerebral levels of lactic acid and FFA, indicating that PNS possess the functions of improving brain tissue energy metabolism and reducing neuronal damage under hypoxia/ischemia. The reduction in abnormal calcium concentration in rat cerebral tissues is more evident, and the therapeutic action of PNS on cerebral ischemia is involved in improving cerebral energy metabolism.

Previous studies have identified two strategies involved in hypoxia-anoxia defense mechanisms: (1) reduction in energy (ATP) turnover and (2) improved energetic efficiency of those metabolic processes, particularly the efficiencies of ATP-producing pathways [34]. Diminishing ATP demand and supply (e.g., reducing consumptive processes) to meet the suppression of energy turnover and maximizing either of the ATP-yielding processes both per mole of oxygen in aerobic pathways and per mole of H^+^ in anaerobic pathways can provide substantial protection against hypoxia-anoxia [34, 35]. The results of the present study indicate that cerebral ischemic rats treated with PNS showed higher levels of ATP and its energy-reserve PCr in brain tissue, very likely the hypoxia defense basis on which PNS-treated mice could survive longer under hypoxic-anoxic conditions (in sealed jar). Because PNS simultaneously reduced the levels of lactic acid and FFA in the brain tissues of cerebral ischemic rats, we speculate that its hypoxia defense ability is unlikely to be achieved by increasing anaerobic ATP supply pathways instead of by reducing ATP turnover [34]. The hypoxia defense ability of PNS is also almost impossible to achieve by increasing aerobic energy pathways because ATP production via oxidative phosphorylation is extremely decreased and even ceases under hypoxia-anoxia conditions. Further studies are necessary to determine how the hypoxia-resistant ability of PNS is achieved under cerebral ischemic conditions.

## 5. Conclusion

In the present study, various experimental animal models were used to investigate the effects of PNS on cerebral ischemia. PNS improved neurobehavioral function under cerebral ischemia conditions, increased hypoxia resistance, and reduced systemic thromboembolism damage. The pharmacological mechanisms underlying the actions of PNS on cerebral ischemia are associated with reduced cerebral pathological damage, thrombolysis, improvement in intracellular Ca^2+^ overload, and cerebral energy metabolism. In particular, the present study provides novel insight that PNS exert antihypoxic action primarily by reducing energy turnover (e.g., ATP consumption) but not by affecting ATP-yielding processes.

## Figures and Tables

**Figure 1:** PNS reduce the cerebral infarction area and improve neurological function in MCAO rats. (a) Representative TTC staining images of the coronal sections of rats in each group after MCAO. (b) Cerebral infarction area ratios of the rats in each group. (c) Results of functional neurobehavioral scoring. PNS: *Panax notoginseng* saponins; MCAO: middle cerebral artery occlusion; SO: sham-operated group; TTC: triphenyl tetrazolium chloride. The data were presented as means ± SD (*n* = 10). Statistical comparisons were evaluated using one-way ANOVA with the Newman–Keuls post hoc test. ∗*P* < 0.05 and ∗∗*P* < 0.01 compared with the MCAO model group.

**Figure 2:** PNS increase the coordination function in cerebral ischemia rats. (a) Average maximum angles at which rats slipped down from an inclined smooth plane. (b) Cerebral index of the four artery blocked rats. PNS: *Panax notoginseng* saponins; SO: sham-operated group. The data were presented as means ± SD (*n* = 10 or 9). Statistical comparisons were evaluated using one-way ANOVA with the Newman–Keuls post hoc test. ^∗∗^*P* < 0.01 compared with the ischemia model group.

**Figure 3:** PNS inhibit acute systemic intravascular thromboembolism induced by collagen-adrenaline in mice. (a) Time from collagen-adrenaline injection to hemiplegia of mice. The results were presented as the percentage of normal mice as a function of time. (b) Number of hemiplegic mice induced by collagen-adrenaline within 15 min. *P* < 0.05 and ^∗∗^*P* < 0.01 (*n* = 12, *χ*^2^ test) compared with the thrombosis model group. (c) Time from collagen-adrenaline injection to the death of mice. The results were presented as the percentage of mice alive as a function of time. (d) Number of dead mice within 5 min. ^∗^*P* < 0.05 (*n* = 12, *χ*^2^ test) compared with the thrombosis model group. PNS: *Panax notoginseng* saponins.

**Figure 4:** PNS inhibit arteriovenous (AV) shunt thrombosis in rats. Thrombosis was formed in common carotid artery-jugular vein blood flow in the bypass, and the inset shows the thrombosis inhibition rate of each PNS-treated group. The data were presented as means ± SD (*n* = 10). Statistical comparisons were evaluated using one-way ANOVA with the Newman–Keuls post hoc test. ^∗∗^*P* < 0.01 compared with the thrombosis model group. PNS: *Panax notoginseng* saponins.

**Figure 5:** PNS prolong the hypoxia tolerance time in mice. The hypoxia tolerance time was recorded from when a mouse was sealed in the jar to its death. The data were presented as means ± SD (*n* = 10). Statistical comparisons were evaluated using one-way ANOVA with the Newman–Keuls post hoc test. ^∗^*P* < 0.05 compared with the hypoxia model group. PNS: *Panax notoginseng* saponins.

**Table 1:** Effects of PNS on brain tissue metabolites in cerebral ischemic rats subjected to four-vessel occlusion.

Group	n	Dose (mg/kg)	Lactic acid (*μ*mol/g)	FFA (*μ*mol/g)	ATP (*μ*mol/g)	Phosphocreatine (*μ*mol/g)	Ca^2+^ (*μ*g/g)
SO	10	9.13 ml	7.60 ± 0.43∗∗	0.036 ± 0.006∗∗	2.87 ± 0.16∗∗	2.21 ± 0.27∗∗	40.88 ± 3.34∗∗
Ischemia model	10	9.13 ml	21.08 ± 1.59	0.091 ± 0.008	0.39 ± 0.09	1.06 ± 0.20	65.83 ± 2.52
Low-dose PNS	10	18.30	20.99 ± 1.39	0.090 ± 0.006	0.40 ± 0.08	1.20 ± 0.16	63.96 ± 3.43
Middle-dose PNS	10	36.50	19.64 ± 1.35	0.082 ± 0.006∗	0.49 ± 0.10∗	1.41 ± 0.12∗∗	59.79 ± 2.65∗∗
High-dose PNS	10	73.00	15.69 ± 1.07∗∗	0.070 ± 0.007∗∗	0.72 ± 0.12∗∗	1.55 ± 0.12∗∗	54.98 ± 3.06∗∗

PNS: *Panax notoginseng* saponins; FFA: free fatty acid; ATP: adenosine triphosphate; SO: sham-operated; data were presented as means ± SD; ∗*P* < 0.05 and ^∗∗^*P* < 0.01 compared with ischemia model.

## Data Availability

The data used to support the findings of this study are available from the corresponding author upon request.
